# Sevoflurane inhibits the progression of ovarian cancer through down-regulating stanniocalcin 1 (STC1)

**DOI:** 10.1186/s12935-019-1062-0

**Published:** 2019-12-16

**Authors:** Chuanfeng Zhang, Baosheng Wang, Xiuqin Wang, Xiugui Sheng, Yongchun Cui

**Affiliations:** 1 Shandong Cancer Hospital Affiliated to Shandong University, Jinan, 250117 China; 2 Shandong Cancer Hospital and Institute, Shandong First Medical University and Shandong Academy of Medical Sciences, Jinan, 250117 China; 3 National Cancer Center/National Clinical Research Center for Cancer/Cancer Hospital and Shenzhen Hospital, Chinese Academy of Medical Sciences and Peking Union Medical College, Shenzhen, 518116 China

**Keywords:** Sevoflurane, Ovarian cancer, Stanniocalcin 1, Growth, Invasion, MMP-9

## Abstract

**Background:**

Ovarian cancer is one of the leading causes of female death worldwide, with a poor prognosis of advanced patients. Sevoflurane, a volatile anesthetic commonly used in clinical operations, has been reported to have anti-cancer activity against some tumors. In the present study, we aimed to investigate the effects of sevoflurane on the progression of ovarian cancer and its potential mechanism.

**Methods:**

The effects of sevoflurane on ovarian cancer cell viability, proliferation, migration, invasion, cell cycle, and apoptosis were determined by functional experiments in vitro. Gelatin zymography assay was performed to examine MMP9 activity. In vivo, sevoflurane was injected into mice of transplantation tumor with SKOV3 cells or with pcDNA-STC1 treated SKOV3 cells.

**Results:**

We found that sevoflurane inhibited the viability of SKOV3 and OVCAR3 cells in a dose-dependent manner, and colony formation assay revealed that sevoflurane inhibited ovarian cancer cell colony-formation abilities. Additionally, sevoflurane could induce cell cycle arrest and promote cell apoptosis in SKOV3 and OVCAR3 cells. Moreover, sevoflurane reduced the migration and invasion abilities of SKOV3 and OVCAR3 cells, as well as the MMP-9 activity. Furthermore, sevoflurane down-regulated the expression of stanniocalcin 1 (STC1), and up-regulation of STC1 could reverse the inhibitory effects of sevoflurane on cell proliferation and invasion. In vivo, sevoflurane significantly inhibited the tumor growth, which was be reversed by STC1 overexpression.

**Conclusion:**

These data reveal an anti-cancer activity of sevoflurane on the growth and invasion of ovarian cancer, which may be through down-regulating STC1. Sevoflurane may serve as a potential anti-cancer agent in ovarian cancer therapy.

## Background

Ovarian cancer is a highly lethal gynecological malignancy and is one of the leading causes of female death, with nearly 239,000 new cases and 152,000 deaths worldwide each year [1]. According to statistics, a woman’s lifetime risk of ovarian cancer is 1/75, and the probability of dying from ovarian cancer is 1/100 [2]. What is more distressing is that most patients are in advanced stage at the time of diagnosis, accompanied by local or distant metastasis, leading to poor prognosis. The overall 5-year relative survival rate of ovarian cancer patients worldwide is generally between 30% and 40% [3]. The 5-year survival rate of advanced patients is only 29%, while that of early patients is 93% [2, 4]. Although the treatment strategies and surgical techniques have been significantly improved, the prognosis of ovarian cancer remains unsatisfactory. The main causes of high mortality and poor prognosis of ovarian cancer are the lack of early diagnosis and resistance to chemotherapy [5, 6]. Therefore, it is necessary to find new targeted agents and strategies for ovarian cancer.

It is well known that surgical resection of tumors is an important method of cancer treatment. Increasing evidences show that anesthetics used in surgical resection also have certain non-anesthetic physiologic effects, which can affect the invasion and migration abilities of tumor cells [7, 8]. Sevoflurane is a volatile anesthetic commonly used in clinical operations. It has been reported that sevoflurane can inhibit the proliferation of colon cancer, laryngeal cancer cells [9, 10] and head and neck squamous cell carcinoma [11], and decrease the migration and invasion abilities of lung cancer [12, 13] and glioma cells [14, 15]. These studies reveal an anti-tumor activity of sevoflurane, suggesting that sevoflurane may be used as a potential target agent for treatment of cancer. However, little is known about the effects of sevoflurane on the proliferation and invasion of ovarian cancer.

In the present study, for the first time, we investigated the effects of sevoflurane on the proliferation and invasion of ovarian cancer cells. Moreover, we revealed the molecular mechanism of sevoflurane underlying its anti-tumor activity in ovarian cancer cells.

## Materials and methods

### Cell culture and treatment

The human ovarian cancer cell lines SKOV3 and OVCAR3 were obtained from the Cell Bank of Chinese Academy of Sciences (Shanghai, China). Cells were routinely grown in DMEM medium supplemented with 10% fetal bovine serum (FBS), 100 U/mL penicillin (Sigma-Aldrich, Germany) and 0.1 mg/mL streptomycin (Sigma-Aldrich). SKOV3 and OVCAR3 cells were cultured in medium supplemented with sevoflurane (Maruishi Pharmaceutical, Japan) in vitro, and DMSO was used as negative control (NC). The STC1 cDNA sequence was cloned into the pcDNA3.1 vector to construct the STC1 expressing plasmid. Cells were transfected with pcDNA3.1-STC1 vector using Lipofectamine 2000 (Invitrogen, USA) to up-regulate the expression of STC1, and the control group was transfected with an empty vector.

### CCK8 assay

Cells were exposed to different concentration of sevoflurane (0.5, 1, 1.5, 2, 2.5, 3, 4, 5, and 6% for SKOV3 cells; 0.5, 1, 1.5, 2, 2.5, 3, 3.5, 4, 4.5, 5, 5.5, 6, 6.5, 8 and 10% for OVCAR3 cells) in a 96-well plate at 37 °C for 24 h. With an addition of cell Counting Kit-8 reagent (10 μL/well; CCK8; Beijing Solarbio Science & Technology, Beijing, China), cells were cultured for 90 min at 37 °C. The absorbance was measured at 450 nm with a Bio-Rad microplate reader (Bio-Rad Laboratories, USA).

### Colony formation assay

SKOV3 and OVCAR3 cells were treated with sevoflurane for 24 h, and grown in 35 mm-plates at a density of 5 × 10^2^/well and cultured in DMEM at 37 °C for about 1 week until the visible colonies were formed. Then, the medium was removed and the colonies were fixed with 4% paraformaldehyde for 30 min followed by staining with 0.1% crystal violet for 30 min. The colonies were counted and photographed.

### Cell cycle analysis

Flow cytometry was performed to assess the effect of sevoflurane on cell cycle distribution. After 24 h treatment with sevoflurane at 37 °C, cells were collected and fixed with 70% pre-cooling ethanol at − 20 °C overnight. After that, cells were stained with propidium iodide (PI) for 30 min in the dark, the cell cycle was analyzed using a flow cytometer (BD FACSC anto II, BD Biosciences, USA). The data was analyzed with BD FACSDiva software (BD Bioscience).

### Cell apoptosis analysis

Annexin V-FITC/PI kit (BD Bioscience) was performed to examine cell apoptosis. SKOV3 and OVCAR3 cells were treated with sevoflurane for 24 h, and cells were collected and stained with 5 μL of Annexin V-FITC for 5 min in the dark and stained with 10 μL of PI at room temperature. The rate of apoptosis in each sample was analyzed using a flow cytometer (BD FACSC anto II) and calculated by BD FACSDiva software.

### Western blot

After being treated with sevoflurane for 48 h, cells were harvested and lysed with RIPA Lysis Buffer (CWBIO, Beijing, China) to extract protein. Then, 20 µg protein of each sample was electrophoresed on 10% SDS-PAGE gel, and transferred onto polyvinylidene fluoride membrane (PVDF; Millipore, Billerica, MA, USA). Subsequently, the members were blocked with 5% dried skimmed milk for 1 h followed by incubation with primary antibodies (dilution, 1:1000; Proteintech Group, IL, USA) at 4 °C overnight. After labelling with horseradish peroxidase (HRP)-conjugated secondary antibodies (dilution, 1:3000; Proteintech Group) for 1 h, the signals were visualized using an Enhanced Chemiluminescence kit (CWBIO). β-tubulin was used as endogenous control, and the relative expression of proteins were normalized to NC.

### Wound-healing assay

A wound-healing assay was performed to assess cell migration ability. About 5 × 10^5^ cells per well were grown in a 6-well plate and cultured for 24 h at 37 °C. Subsequently, cells were scraped with pipette tips to generate a straight-line “wound”. After then cells were treated with sevoflurane for 24 h at 37 °C. Cells were photographed and the wound closure was analyzed quantitatively using ImageJ software (National Institutes of Health, USA).

### Transwell assay

Cell migration and invasion abilities were examined using the Transwell assay. Transwell chamber (Millipore, MA, USA) were coated with Matrigel (BD Bioscience, CA, USA) for cell invasion assay. SKOV3 and OVCAR3 cells were treated with sevoflurane for 24 h and suspended in serum-free medium at 1 × 10^6^ cells/mL. 100 µL of cell suspensions were added into the upper inserts, and 700 µL of complete medium supplemented with 20% FBS was added to the lower chamber as the chemo attractant. After incubation for 24 h, the invaded cells were fixed with 4% paraformaldehyde for 30 min prior to stain with 0.1% crystal violet for 20 min. The migration assay was performed in the same manner as the invasion assay, except that Matrigel was not required. The invaded and migrated cells were imaged (magnification, 100×) and counted under the light microscope.

### Gelatin zymography assay

Gelatin zymography assay was used to examine the effect of sevoflurane on MMP-9 activity. SKOV3 and OVCAR3 cells were cultured for 48 h at 37 °C in serum-free medium supplemented with sevoflurane. After that, cell culture supernatants were collected and electrophoresed on a 10% SDS-PAGE containing 0.5 mg/mL gelatin. The gel was eluted two times in the eluent (2.5%Triton X-100, 50 mM Tris–HCl, 5 Mm CaCl_2_, pH7.6), then washed in the rinsing solution without Triton X-100 and incubated with the incubation solution (50 mM Tris–HCl, 5 Mm CaCl_2_, 0.02% Brij-35, pH 7.6) for 42 h at 37 °C. After incubation, the gel was stained with 0.05% Coomassie Blue R250 for 4 h prior to decolorization at room temperature. The band of MMP-9 was scanned using an Image Scanner (Amersham, USA) and analyzed by ImageQuant TL V2003 software.

### Animal model

The animal experiments in this study were performed according to the guidelines for the care and use of laboratory animals and approved by Shandong Cancer Hospital Affiliated to Shandong University. The transplanted tumor model was established with reference to Zhang et al. [16]. SKOV3 cells were prepared with or without transfection of pcDNA3.1-STC1. Eighteen BALB/c-Nude mice (female, 4–6 weeks old; Shanghai SLAC Laboratory Animal Co., Ltd.) were randomly divided into three groups: Group 1 and Group 2 were injected subcutaneously with 5 × 10^5^ SKOV3 cells into the right armpit of mice; Group 3: mice were injected with SKOV3 cells transfected with pcDNA3.1-STC1. After 7 days of feeding, we dissolved the sevoflurane (50 mg/kg) in 0.5 mL of soybean oil and injected into Group 2 and Group 3 mice for 3 weeks (once a day), Group 1 was injected with the same volume of soybean oil as control. Tumor size was measured every 4 days, and the tumor size was measured after mice sacrifice.

### Statistical analysis

All data were performed as mean ± SD from triplicate independent experiments and statistically analyzed using GraphPad Prism 7.0 (GraphPad, CA, USA). Differences between groups were analyzed using the student’s t test or one-way ANOVA, and P < 0.05 was considered statistically significant.

## Results

### Sevoflurane inhibits the proliferation of ovarian cancer cells

To investigate the cytotoxicity of sevoflurane to ovarian cancer, SKOV3 and OVCAR3 cells were treated with different concentration of sevoflurane. As shown in Fig. 1a, after 24 h of treatment, sevoflurane inhibited cell viability in a dose-dependent manner in SKOV3 cells, and the IC_50_ of sevoflurane for SKOV3 cells was 1.598%. Similarly, a decrease in cell viability caused by different concentrations of sevoflurane was observed in OVCAR3 cells, whereas in OVCAR3 cells, the IC_50_ of sevoflurane was 1.350% (Fig. 1b). Therefore, in the following experiments, SKOV3 cells were treated with 0.95% of sevoflurane, and OVCAR3 cells were treated with 0.8% of sevoflurane for its appropriate effect. The colony formation assay was performed to further assess the growth-inhibitory effect of sevoflurane on ovarian cancer cells. As expected, in comparison with NC group, sevoflurane significantly suppressed colony-formation abilities of SKOV3 and OVCAR3 cells (Fig. 1c).

**Fig. 1:** Sevoflurane inhibits the viability and colony-formation ability of ovarian cancer cells. **a**, **b** SKOV3 (**a**) and OVCAR3 (**b**) cells were treated with different concentrations of sevoflurane for 24 h, CCK8 assay was performed to examine cell viability. **c** After being treated with sevoflurane, colony formation assay was performed. The data were expressed as the mean ± SD from three independent experiments. *P < 0.05, **P < 0.01 vs. the negative control group

### Sevoflurane induces cell cycle arrest in ovarian cancer cells

Given the inhibitory effect of sevoflurane on cell proliferation of ovarian cancer, we examined its effect on cell cycle distribution by flow cytometry. The results showed that the percentage of cells in the G0/G1 phase was significantly increased in SKOV3 cells exposed to sevoflurane, and the proportions of cells in the S phase was decreased compared with NC group (Fig. 2a). In OVCAR3 cells, the results were similar, and the proportion of cells in the G0/G1 phase was also significantly increased, and the proportions of cells in the S and G2/M phases were both decreased (Fig. 2a). Moreover, we examined the expression of cell cycle-related proteins using western blot analysis. Our data showed that sevoflurane caused a significant decrease in the expression level of Cyclin D1 and CDK4 in SKOV3 and OVCAR3 cells (Fig. 2b). Collectively, these data suggest that sevoflurane could induce cell cycle arrest at the G0/G1 phase in SKOV3 and OVCAR3 cells via down-regulating the expression of Cyclin D1 and CDK4.

**Fig. 2:** Sevoflurane induces cell cycle arrest in ovarian cancer cells. **a** SKOV3 and OVCAR3 cells were treated with sevoflurane for 24 h, the cell cycle distribution was analysed by flow cytometry. **b** Cells were incubated with sevoflurane for 48 h, the expression of Cyclin D1 and CDK4 was examined using western blot analysis. The data were expressed as the mean ± SD from three independent experiments. *P < 0.05 vs. the negative control group

### Sevoflurane promotes cell apoptosis in ovarian cancer cells

The effect of sevoflurane on cell apoptosis in ovarian cancer was evaluated using PI-Annexin V double staining. Our data showed that, in comparison with NC group, sevoflurane obviously promoted the rate of apoptosis in both SKOV3 and OVCAR3 cells (Fig. 3a). Changes in expression levels of apoptosis-related proteins after exposure to sevoflurane were examined by western blot to further investigate the mechanism underlying the inducted apoptosis. As indicated in Fig. 3b, the expression of anti-apoptosis protein Bcl-2 was significantly down-regulated by sevoflurane in both SKOV3 and OVCAR3 cells, while the expression of pro-apoptosis proteins Bax and cleaved Caspase3 was up-regulated in sevoflurane-treated group (Fig. 3b). These data indicate that sevoflurane induces cell apoptosis in ovarian cancer cells through regulating the Bcl-2/Bax axis and Caspase activity.

**Fig. 3:** Sevoflurane promotes cell apoptosis in ovarian cancer cells. **a** Flow cytometry was used to detect the rate of apoptosis in SKOV3 and OVCAR3 cells exposed to sevoflurane for 24 h. **b** After 48 h of incubation with sevoflurane, the expression of apoptosis-related proteins (Bcl-2, Bax and cleaved Caspase3) was detect by western blot analysis. The data were expressed as the mean ± SD from three independent experiments. *P < 0.05, **P < 0.01 vs. the negative control group

### Sevoflurane inhibits the migration and invasion abilities of ovarian cancer cells

As shown in Fig. 4a, SKOV3 and OVCAR3 cells treated with sevoflurane exhibited significant depression in migration compared with NC group. Additionally, the Transwell migration assay reveled similar results that sevoflurane significantly inhibited migration ability of SKOV3 and OVCAR3 cells (Fig. 4b). Moreover, sevoflurane inhibited the invasion ability of SKOV3 and OVCAR3 cells that the number of invading cells in the sevoflurane-treated group was much lower compared with NC group (Fig. 4c). Taken together, these results reveal an anti-motility activity of sevoflurane in ovarian cancer.

**Fig. 4:** Sevoflurane reduces the migration and invasion abilities of ovarian cancer cells. **a** Images and wound closure percentage of SKOV3 and OVCAR3 cells for 24 h after sevoflurane treatment. **b**, **c** Transwell assays were used to detect cell migration (**b**) and invasion (**c**) in sevoflurane-treated SKOV3 and OVCAR3 cells. The data were expressed as the mean ± SD from three independent experiments. *P < 0.05 vs. the negative control group

### Sevoflurane inhibits the Akt/mTOR/p70S6k signaling pathway and MMP-9 activity

In view of the pivotal role of Akt/mTOR signaling pathway in the regulation of cell proliferation and survival, changes in the expression of key components of Akt/mTOR pathway were detected under sevoflurane treatment. As indicated by Western blot, the expression of total Akt and mTOR did not been affected by sevoflurane in both SKOV3 and OVCAR3 cells, while the phosphorylation levels of Akt (p-Akt) and mTOR (p-mTOR) were significantly decreased (Fig. 5a). The expression of p70S6k was also down-regulated by sevoflurane treatment (Fig. 5a). In addition, we found that the activity of MMP-9, a key regulator involved in invasion process, was significantly diminished in SKOV3 and OVCAR3 cells treated with sevoflurane (Fig. 5b).

**Fig. 5:** Sevoflurane inhibits the Akt/mTOR signaling pathway and MMP-9 activity. **a** SKOV3 and OVCAR3 cells were treated with sevoflurane for 48 h, the effects of sevoflurane on Akt/mTOR signaling pathway were analyzed by western blot assay. **b** Gelatin zymography assay was used to examine the effect of sevoflurane on MMP-9 activity. The data were expressed as the mean ± SD from three independent experiments. *P < 0.05 vs. the negative control group

### Sevoflurane inhibits cell proliferation and invasion by down-regulating stanniocalcin 1 (STC1)

To further elucidate the potential mechanisms underlying the anti- growth and –invasion activity of sevoflurane in ovarian cancer, RNA-Seq by PossionDis was performed to determine significantly differential expressed genes (|log_2_ fold change| > 1 and Q value < 0.001) in sevoflurane-treated cells. The data showed that the expression of STC1 was significantly down-regulated by sevoflurane, which was further confirmed by the results of western blot (Fig. 6a). In addition, transfection with pcDNA3.1-STC1 reversed the inhibitory effect of sevoflurane on the expression of STC1 in both SKOV3 and OVCAR3 cells compared to those after sevoflurane treatment alone (Fig. 6a). Therefore, STC1 might be a target gene for sevoflurane.

**Fig. 6:** Sevoflurane inhibits cell proliferation and invasion in ovarian cancer by down-regulating STC1. SKOV3 and OVCAR3 cells were transfected with pcDNA3.1-STC1 or pcDNA3.1-vector and were then co-treated with sevoflurane. **a** After 48 h of treatment, western blot assay was performed to examine the expression of STC1. **b**, **c** After 24 h of treatment, CCK8 assay was used to examine cell viability of SKOV3 (**b**) and OVCAR3 (**c**) cells. **d** Cell migration and invasion were assessed by Transwell assay. **e** Quantitative analysis of transwell results. **f** The activity of MMP-9 was examined by gelatin zymography assay. The data were expressed as the mean ± SD from three independent experiments. *P < 0.05, **P < 0.01 vs. the negative control group

STC1 has been revealed to be up-regulated in ovarian cancer and involved in tumor progression [17]. We suspected that STC1 may be involved the effect of sevoflurane on proliferation, migration and invasion of ovarian cancer cells. Our data showed that up-regulation of STC1 reversed the suppression in cell viability caused by sevoflurane in a time-dependent manner in SKOV3 cells (Fig. 6b). Similar results were observed in OVCAR3 cells (Fig. 6c). Next, a Transwell assay was used to assess cell migration and invasion. As shown in Fig. 6d, e, the depression in the migration ability induced by sevoflurane was significantly rescued by the up-regulation of STC1 in both SKOV3 and OVCAR3 cells. Moreover, the inhibitory effect of sevoflurane on cell invasion was also reversed by the presence of STC1 in SKOV3 and OVCAR3 cells (Fig. 6d, e). Furthermore, up-regulation of STC1 also reversed the activity of MMP-9 in sevoflurane-treated cells (Fig. 6f).

### Sevoflurane reduces the growth of tumor by regulating STC1 in vivo

The model of transplantation tumor of SKOV3 cells in nude mice was established. As shown in Fig. 7a, b, we observed that the injection of 50 ng/kg sevoflurane significantly reduced the tumor volume compared with the NC group, while the anti-tumor effect of sevoflurane could be partly reversed by up-regulation of STC1.

**Fig. 7:** Sevoflurane reduces tumor volume in SKOV3 cell transplanted tumor mice. SKOV3 cells with or without transfection of pcDNA3.1-STC1 were injected into the nude mice for 7 days. Mice were injected of 50 ng/kg sevoflurane (dissolved into 0.5 mL soybean oil) or 0.5 mL soybean oil for 3 weeks. After the mice were sacrificed, the tumor was dissected (**a**) and the tumor volume was measured (**b**). *P < 0.05 vs. the negative control group, ^#^P < 0.05 vs. the sevoflurane treatment

## Discussion

It has been reported that anesthesia and anesthesia techniques may influence the progression of cancer after surgery [7, 18]. Sevoflurane has been revealed to inhibit cell migration and invasion in lung cancer and glioma cells [12–15]. In this study, we firstly demonstrated that sevoflurane significantly inhibited the proliferation of ovarian cancer SKOV3 and OVCAR3 cells in a dose-dependent manner, and reduced cell migration and invasion abilities, as well as inhibited tumor growth in vivo. Moreover, treatment with sevoflurane induced cell cycle arrest and promoted cell apoptosis in SKOV3 and OVCAR3 cells. Collectively, these results suggest that sevoflurane might serve as an anti-tumor agent for therapy of ovarian cancer.

It is well known that inducing cell cycle arrest and promoting apoptosis are two effective approaches to inhibit cell growth. Normal cell cycle process is the key mechanism for cell proliferation, and cancer cells are commonly characterized by cell cycle dysregulation [19, 20]. Blocking cell cycle is also one of the mechanisms of many anti-cancer agents [21–23]. It has been reported that sevoflurane induces cell cycle arrest at G1 phase in breast cancer cells [24]. In our study, we found that the proportion of cells in the G0/G1 phase was significantly increased in sevoflurane-treated group, the proportion in the S phase was accordingly decreased (Fig. 2), denoting a remarked cell cycle arrest at G0/G1 phase induced by sevoflurane in ovarian cancer cells, which was consistent with previous study [24]. Moreover, the expression of Cyclin D1 and CDK4, the key regulators in promoting cell transition from G1 phase to S phase, was significantly down-regulated by sevoflurane. Collectively, sevoflurane arrests cell cycle in the G0/G1 phase through down-regulating Cyclin D1/CDK4, resulting in the inhibition of cell proliferation.

Promoting tumor cell apoptosis is one of the important features of cytotoxic anti-tumor agents [25–27]. In the current study, our results from flow cytometry suggested that sevoflurane promoted the rate of apoptosis in SKOV3 and OVCAR3 cells (Fig. 3). Bcl-2 and caspase families are key regulators involved in apoptosis process [27, 28]. We observed that the expression of Bcl-2 was significantly up-regulated by sevoflurane, whereas the expression of Bax and cleaved Caspase3 was down-regulated, indicating that sevoflurane promotes cell apoptosis in ovarian cancer through regulating the Bcl-2/Bax axis and Caspase cascade. Yang et al. [11] report that sevoflurane induces apoptosis and suppresses the expression of Bcl-2 in head and neck cancer cell lines FaDu and CAL-27. Taken together, these results indicates that sevoflurane may exert its anti-growth effect through triggering cell cycle arrest and inducing apoptosis in ovarian cancer.

The Akt/mTOR signaling pathway has been implicated in cancer development, and is frequently aberrant activated in cancers. Akt/mTOR signaling pathway has been proved to play pivotal roles in the regulation of cell proliferation, cell cycle and apoptosis [29, 30]. The suppression of the Akt/mTOR signaling has been shown to be an effective strategy to the treatment of cancers and is the mechanism for the activity of many anti-tumor agents [31, 32]. Our study demonstrated that sevoflurane could reduce the phosphorylation of Akt and mTOR in SKOV3 and OVCAR3 cells (Fig. 5). Additionally, the expression of p70S6k, the target of mTOR, was accordingly down-regulated by sevoflurane. In head and neck cancer cells, sevoflurane is revealed to inhibit the phosphorylation of Akt [11], which is consistent with our results in ovarian cancer. Liang et al. [12] reveal that sevoflurane inhibits the migration and invasion abilities of A549 cells through inhibiting p38 MAPK signaling pathway and the activities of MMP-2 and MMP-9. Hurmath et al. [15] find that sevoflurane suppresses the migration of U87MG glioma cells by attenuating the activity of MMP-2. Herein, we observed that sevoflurane significantly attenuated the activity of MMP-9 in SKOV3 and OVCAR3 cells. In combination with the above studies, we suggest that the Akt/mTOR signaling pathway and MMP-9 might be implicated in the anti-tumor activity of sevoflurane.

Further assays were performed to investigate the molecular mechanism underlying the anti-tumor activity of sevoflurane in ovarian cancer. From high-throughput sequencing and western blot analysis, we found that the expression of STC1 was significantly down-regulated in sevoflurane-treated cells. STC1, a secreted glycoprotein, has been reported to be involved in several pathologies, including angiogenesis and inflammation [33–35]. Emerging evidences have revealed that STC1 is implicated in carcinogenesis and the progression of mangy types of cancer, including but not limited to colorectal, breast, hepatocellular carcinoma, cervical, and ovarian cancer [17, 36–39]. Liu et al. [17] has reported that STC1 is up-regulated in ovarian cancer tissues, cell lines and serum from patients, its overexpression could promote cell proliferation, migration and tumor growth in mice model. Moreover, knockdown of STC1 could arrest cell cycle in G0/G1 phase and promote apoptosis in SKOV3 cells [17], suggesting an oncogenic role of STC1 in ovarian cancer. In the current study, the suppression in cell proliferation, migration and invasion caused by sevoflurane was significantly reversed by the up-regulation of STC1 in SKOV3 and OVCAR3 cells, as well as MMP-9 activity (Fig. 6). Further, we observed that the inhibition of sevoflurane in tumor growth was reserved by up-regulation of STC1. These results indicate that sevoflurane may exert the anti-tumor activity through targeting STC1 in ovarian cancer.

## Conclusion

In summary, for the first time, our data demonstrate sevoflurane inhibits cell proliferation, migration and invasion and induces cell cycle arrest and apoptosis in ovarian cancer cells through targeting STC1. The Akt/mTOR signaling pathway may be implicated in the anti-tumor activity of sevoflurane. This study provides evidence that sevoflurane might represent a potential novel targeted agent in the treatment of ovarian cancer. Further study is needed to investigate the anti-tumor activity of sevoflurane in mice model and its deeper molecular mechanism.

## Data Availability

The data supporting the conclusions of this paper are included within the manuscript.

## Abbreviations

Akt: protein kinase B
CCK8: cell counting kit-8 reagent
FBS: fetal bovine serum
GEPIA: Gene Expression Profiling Interactive Analysis
mTOR: mammalian target of rapamycin
STC1: stanniocalcin 1
